RETRACTED

# Epidemiological Features of COVID-19 in Makkah City: A Retrospective Data Analysis

**DOI:** 10.1155/2022/8301490

**Published:** 2022-02-24

**Authors:** Atif Asghar, Majid Bamaga, Asim Khogeer, Ibrahim Abd El-Rahim, Bassam Mashat, Hamza Assaggaf, Omar Ahmed

**Affiliations:** ^1^Department of Environmental and Health Research, The Custodian of The Two Holy Mosques Institute of Hajj and Umrah Research, Umm Al-Qura University, P.O. Box: 6287, Makkah, Saudi Arabia; ^2^Plan and Research Department, General Directorate of Health Affairs Makkah Region, MOH, Saudi Arabia; ^3^Department of Laboratory Medicine, Faculty of Applied Medical Sciences, Umm Al-Qura University, Makkah 24381, Saudi Arabia

## Abstract

**Background:**

Coronavirus disease 2019 (COVID-19) is continuing to circulate and change, affecting billions of people worldwide and leading to increased mortality rates, especially in the Holy City of Makkah, Kingdom of Saudi Arabia (KSA). This study was aimed at investigating the epidemiological features of COVID-19 in Makkah City, KSA.

**Methods:**

A retrospective analysis was conducted to investigate the prevalence of COVID-19 and the association between the severity and mortality of COVID-19 with demographic factors and comorbidities.

**Results:**

Among 4,742 COVID-19 patients, the incidence rate observed in males was 66.7%, and 69.7% were from Al-Noor Specialized Hospital. The highest incidence rate (25.2%) was found in the age group > 60 years old, followed by the age group 51-60 years (21.8%). Furthermore, the highest frequency was observed in patients from Saudi Arabia (36.8%), followed by patients from Myanmar (14.7%) and Bangladesh (9.4%). The overall frequency of COVID-19 severity and death was 20.3% and 11.6%, respectively. Body mass index analysis showed that 1% of the patients were underweight, while 9.2% were overweight and 4.4% were obese. In addition, 9.6% had diabetes, 6.9% had hypertension, 1.1% had heart disease, and 2.2% had other chronic diseases.

**Conclusion:**

The study concluded that the overall percentages of severe COVID-19 (intensive care unit) cases and deaths in Makkah City, KSA, were 20.3% and 11.6%, respectively, and there was a higher incidence in male patients. The severity of infection was shown to have a strong significant correlation with different chronic diseases, nationality, body mass index, death rate (mortality), heart disease, and length of hospital stay (*P* < 0.05). Despite these findings, more studies are needed to explain the underlying mechanisms that influence the overall health status of patients with specific characteristics and comorbidities.

## 1. Introduction

After nearly 2 years (December 2019 to December 2021), coronavirus disease 2019 (COVID-19) continues to circulate and change widely. It has affected more than 330 million people and has led to the death of more than 5 million people. Furthermore, common disparities among infected persons play an essential role in the severity of the illness due to severe acute respiratory syndrome coronavirus 2 (SARS-CoV-2) infection. In particular, certain health conditions and demographic factors increase the risk of developing a severe COVID-19 infection and may aggressively affect infection outcomes [1–3]. As of August 15, 2020, the COVID-19 outbreak had exceeded 530,000 confirmed cases in the Kingdom of Saudi Arabia (KSA), and almost all regions and cities were affected. Current statistical reports show that the Holy City of Makkah is the third highest city in the KSA regarding COVID-19-confirmed cases [4].

RETRACTED

The spread of SARS-CoV-2 infection is detrimental, given its association with several parameters, including age and other underlying conditions [5, 6]. A previous study found that patients with underlying health conditions carry a significantly higher risk of infection than healthy individuals [7]. Furthermore, a higher number of deaths have been linked to comorbidities, including cardiovascular disease (CVD) hypertension, asthma, pulmonary diseases, diabetes, cancer, and ethnicity and racial variations [8–22].

In particular, hypertensive patients carry a 3.48-fold increased risk of dying due to SARS-CoV-2 infection. Thus, hypertension can significantly increase the fatality rate among infected individuals [8]. Since health perturbations and various underlying conditions increase the implications of the infection, they predispose infected patients to become more vulnerable. A vulnerable individual's level of immunity and chronic medical conditions also predispose them to becoming infected with the virus [10]. These different parameters increase an individual's risk of developing severe respiratory infections with low oxygen levels and pneumonia, which can lead to a high fatality rate [11, 12]. Adams et al. reported that 45.4% of adults in the USA have a higher risk of developing COVID-19 complications due to hypertension, asthma, pulmonary diseases, CVD, diabetes, and cancer [13]. Consequently, different underlying medical conditions play a major role in worsening the severity of COVID-19 outcomes and increasing the possibility of fatality. According to the Centers for Disease Control and Prevention (CDC) reports, these conditions include cancer, chronic kidney diseases, chronic obstructive pulmonary disease (COPD), immunocompromise, heart conditions, pregnancy, liver disease, sickle cell anemia, and cystic fibrosis. In addition to underlying health diseases, certain demographic factors such as sex and age have also been found to be significantly correlated with infection outcomes [23–26]. Moreover, obesity and hospitalization are strongly correlated with health deterioration [27, 28]. Older patients have been found to be more severely affected by infection, and health deterioration has been linked to further complications [24]. According to recent studies, the risk of severe illness from COVID-19 increases with age [6, 25]. Thus, older adults are at a higher risk of contracting COVID-19 and show severe health deterioration. Another study also found that older populations are significantly affected by the disease and that the infection outcomes and disease prognosis are worse in older patients [26]. In line with these findings, adults aged 65 years and older account for 8 out of 10 COVID-19-related deaths in the USA [17]. In China, in-hospital deaths due to COVID-19 have also been shown to increase with age [6]. Furthermore, obesity is regarded as one of the most significant conditions affecting the severity of COVID-19 and exponentially increases the total number of deaths [16].

RETRACTED

Makkah is the holiest city in Islam; approximately 3 million people from all over the world journey to the city each year to perform the Hajj pilgrimage and Umrah visits. The Hajj pilgrimage to Makkah is considered a planned mass gathering because of the attendance of a large number of people at a specific place for a finite time. One of the main problems regarding mass gatherings, especially pilgrimage events such as Hajj, is the dissemination of infectious diseases. Hence, the severity of illness, health conditions, and demographic factors need to be investigated. Since the emergence of COVID-19, the allowed number of pilgrims in Makkah has decreased substantially, and only a limited number of local pilgrims could perform Hajj in 2020. The present study identified epidemiological features of this disease in Makkah City and raised awareness of the risk and predisposing factors that heavily affect the outcomes of the infection. In particular, this study investigated the epidemiological features of COVID-19 and the associations between severity and mortality with demographic factors and comorbidities for cases in Makkah City, KSA.

## 2. Materials and Methods

### 2.1. Study Population and Design

A multicenter retrospective study was conducted using the Ministry of Health (MOH) registered data for COVID-19 patients who were admitted to a hospital in the city of Makkah from February 1, 2020, to April 30, 2021. The data were collected from five tertiary hospitals with diverse patient populations: King Abdulaziz Hospital (KAH), King Faisal Hospital (KFH), Heraa General Hospital (HGH), Maternity Hospital (MH), and Al-Noor Specialized Hospital (NSH). The study's sample was composed of 4,742 patients who were residents of the holy city of Makkah, KSA, and were registered in the MOH database (electronic medical record [EMR]) for the duration of the period from February 1, 2020, to April 30, 2021. The inclusion criteria were COVID-19 positive as a result of a real-time polymerase chain reaction (RT-PCR) test and were admitted to a Makkah hospital during the study period. Patients who lived outside Makkah City and those who had a negative RT-PCR test were excluded from the study. The study was approved by the Institutional Review Board of the Directorate of Health Affairs (DHA) in the Makkah region, IRB No. H-02-K-076-0920-372, dated in 04.10.2020.

RETRACTED

### 2.2. Data Collection

We extracted all positive SARS-CoV-2 data from the EMR system from each of the targeted hospitals included in this study. A systematic plan was performed during data collection to extract relevant information that was consistent with our targeted population. The variables included the following demographic data, comorbidities, and health-related conditions: gender, age (<20, 21–30, 31–40, 41–50, 51–60, and >60 years), nationality, body mass index (BMI; underweight [<18.5 kg/m^2^], normal [18.5–25 kg/m^2^], overweight [25–30 kg/m^2^], and obese [>30 kg/m^2^]), length of stay in hospital (LOSh), intensive care unit (ICU), patient's status (died, discharged, unknown), and history of chronic diseases.

### 2.3. Statistical Analyses

To identify which variable and severity relationships are moderated by demographic factors, comorbidities, or chronic diseases, we conducted a multicenter retrospective analysis using the Statistical Package for Social Sciences (SPSS version 25; IBM Corp., Armonk, NY).

Baseline clinical characteristics were calculated and presented as frequencies and percentages. Categorical variables with normal distribution were reported as frequencies and percentages and were compared using the chi-square test. Differences were considered statistically significant at *P* values ≤ 0.05.

## 3. Results

The study demonstrated the demographic characteristics and health conditions of a total of 4,742 COVID-19 patients (Table 1). The sample of the reviewed cases comprised 3,162 (66.7%) male patients and 1,580 (33.3%) female patients (Figure 1). Of the five hospitals, NSH treated the most patients (3,307; 69.7%), whereas 552 (11.6%) patients were treated at KAH, 431 (9.1%) were treated at HGH, 301 (6.3%) were treated at KFH, and 151 (3.3%) were treated at MH (Figure 1). The highest rate of incidence (25.2%, *n* = 1,197) was found in the group of patients aged >60 years, followed by those aged 51–60 years (21.8%, *n* = 1,034), and the lowest incidence rate was identified in the group equal to or less than 20 years old (4.3%, *n* = 205), as shown in Table 1. Regarding the nationalities of the reviewed cases, patients from Saudi Arabia had the highest frequency (36.8%, *n* = 1,743), followed by patients from Myanmar (14.7%, *n* = 698) and Bangladesh (9.4%, *n* = 447). The overall number of ICU-admitted patients (severely ill) was 961 (20.3%), while 3,781 (79.7%) patients had no severe illness.

RETRACTED

The BMIs of 1,236 patients were reviewed. The analysis showed that 48 (1%) of the patients were underweight (<18.5 kg/m^2^), 544 (11.5%) were normal (18.5–25 kg/m^2^), 437 (9.2%) were overweight (25–30 kg/m^2^), and 207 (4.4%) were obese (>30 kg/m^2^).

Regarding patient status, 552 (11.6%) of the patients died, 3,401 (71.7%) recovered, and 789 (16.6%) were still admitted at the end of the study period. Of the 4,742 reviewed cases, 455 (9.6%) had diabetes, 328 (6.9%) had hypertension, 51 (1.1%) had heart diseases, and 102 (2.2%) had other chronic diseases (Table 1, Figure 1).

Table 2 shows the various degrees of association between the separately analyzed variables. The findings revealed that COVID-19 severity (ICU admission) was significantly associated with nationality, BMI, death rate (mortality), heart disease, and LOSh (*P* < 0.05). The length of a patient's stay in a hospital was found to be significantly associated with nationality, BMI, COVID-19 severity (ICU admission), death rate (mortality), diabetes, hypertension, kidney diseases, and LOSh (*P* < 0.05). The COVID-19 death rate (mortality) was found to be significantly associated with sex, age, nationality, BMI, diabetes, hypertension, heart disease, and LOSh (*P* < 0.05).

## 4. Discussion

This study investigated various demographic parameters and health conditions of illness due to SARS-CoV-2 infection. The results showed that the majority of cases were collected from the NSH (69.7%) and KAH (11.6%; Figure 1). The Emergency Department of NSH provides health care for millions of people, especially during Hajj (pilgrimage) events. In a similar study conducted in Makkah, NSH demonstrated a high incidence of COVID-19 during the year of the pandemic [29]. In this study, we report that the overall percentage of patients with severe illness from COVID-19 from February 1, 2020, to April 30, 2021, was 20.3%, which represents the cases that required ICU admission. A similar study conducted outside the KSA at a regional medical center reported that the number of COVID-19 patients admitted to ICU was 31% [30]. Generally, an elevated number of ICU admissions in the wake of COVID-19 has been reported [31–33].

RETRACTED

This study showed that the majority of patients (66.7%) were men, while only 33.3% of them were women. In addition, a strong correlation was noted between male sex and a lower chance of recovery, more severe illness, and mortality. It was also reported that men had a relatively higher percentage of infection than women [23]. Gender-based biological variations have been reported to have a profound effect on the COVID-19 outcomes [34]. Such variations were found to be largely tied to the level of immune responses to viral confrontation and elimination; in line with these findings, the reported deaths were significantly higher in men than in women [35]. The analyses of the present study showed a significant association between gender differences and mortality (*P* < 0.05). Although the number of males admitted to the ICU was higher than the number of females, the association was statistically insignificant for gender and ICU admission (Table 2; *P* = 0.21). Likewise, the association between gender and LOS (hospital or ICU) was also statistically insignificant (*P* = 0.78). Many reports have shown that men have a relatively higher percentage of infections than women [3, 36–39]. In addition, a strong correlation was noted between a lower chance of recovery, more severe illness, and male mortality [23]. It was observed that the disease has a clustering onset, inducing respiratory distress with acute pneumonia, and older males with comorbidities are more affected [40].

Our data showed that the percentage of COVID-19 cases increased with age (Table 1). While patients younger than 20 years of age had the lowest prevalence of infection (4.3%), patients older than 60 years had the highest prevalence (25.2%). This relationship is consistent with the age-related severity of infection. Furthermore, patients over 60 years old represented the majority of ICU cases (*P* < 0.05). Thus, the age factor is significantly associated with the severity of COVID-19 and the overall number of deaths. The literature has demonstrated that infected individuals over 60 years old, as well as patients with comorbidities, suffer from a high country-specific crude case fatality rate (CFR) [41, 42]. In Italy, the CFR increased with age. It was less than 1% in patients under 50 years of age and 1.3%–3.6% in patients aged 50–69 years. It was found to range from 8.0% to 12.8% in patients aged 70–79 years and 14.8%–20.2% in patients over 80 years old [26]. Moreover, different studies have reported that patients aged 40–60 years are more susceptible to infection [43], which is in contrast to our findings. In agreement with our findings, Argenziano et al. reported that the infection frequencies were predominant in patients over 60 years old, which was more pronounced in critical care units [14]. Moreover, it has been documented that the number of deaths in the ICU is primarily associated with elderly patients, since severe complications are attributed to different risk factors, including age [44–46]. Furthermore, the nationalities of all reviewed cases show that patients from Saudi Arabia presented the highest frequency (36.8%), followed by patients from Myanmar (14.7%) and Bangladesh (9.4%). A significant association between ICU admission and death was also found in relation to nationality (*P* < 0.05).

RETRACTED

The analysis of BMI showed that 1% of the patients were underweight, 9.2% were overweight, and 4.4% were obese (Figure 1). Obesity is considered another risk factor for contracting SARS-CoV-2, which may result in an increased severity of the illness and lead to death. Analyses of similar studies of BMI correlation in a cohort of COVID-19 patients have shown that 15.8% of the patients died and 88.2% of the patients had a BMI > 25 kg/m^2^ [47, 48]. This relationship may be attributed to the fact that metabolic imbalance in patients with high BMI influences the proinflammatory response, which plays an essential role in viral confrontation [49].

Regarding the mortality rate, the present study found that 11.6% of patients died while 71.7% recovered. A similar study conducted in 11 countries in Asia, Europe, and North America on patients who had COVID-19 found that 24.7% of the patients died in the ICU, while 4% died without ICU admission [50]. Approximately 9.6% of the studied cases in this study had diabetes, 6.9% had hypertension, 1.1% had heart diseases, and 2.2% had other chronic diseases. Moreover, in this study, we found a strong significant correlation between different chronic diseases and the severity of infection. Many studies have also documented that chronic medical conditions affect the severity and complications of infection. For example, hypertension has been reported to account for 60.7%–72.6% of ICU admitted cases, while diabetes accounts for 36.6%–49.2%, and heart diseases account for 8.7%–17.1% [14]. Another study found that patients suffering from chronic conditions had a significantly higher risk of infection than healthy individuals and that 63% of deaths were linked to comorbidities, including CVD and other underlying health complications [7]. Different studies have also found that hypertension, diabetes, and CVD are separately correlated with the severity of COVID-19 [8, 9].

RETRACTED

We faced many challenges during the study, which were mainly related to the relatively small sample size compared to international studies. In addition, different hospitals in Makkah have different data storage methods. We also faced some difficulties related to incomplete demographic data and the investigation findings of some patients. Moreover, it was difficult to determine the actual rates at which positive cases occurred per hospital.

## 5. Conclusions

The study concluded that the overall percentage of severe COVID-19 (ICU) cases and deaths in Makkah City, KSA, were 20.3% and 11.6%, respectively, and there was a higher incidence in male patients. Furthermore, our data showed that the percentage of COVID-19 cases significantly increased with age. A strong significant correlation was observed between infection severity and different chronic diseases, nationality, body mass index, death rate (mortality), heart disease, and length of hospital stay. However, the implications of these findings may help to control COVID-19 in Makkah society including both citizens and pilgrims. Despite these findings, more studies are needed to explain the underlying mechanisms that influence the overall health status of patients with specific characteristics and comorbidities.

## Figures and Tables

**Figure 1:** Demographical characteristics and health conditions for COVID-19 patients.

**Table 1:** Demographical characteristics and frequency of COVID-19 patients (*n* = 4,742).

Variable	Frequency (*n*)	Percent (%)
*Hospital*		
King Abdulaziz Hospital	552	11.6
King Faisal Hospital	301	6.3
Heraa General Hospital	431	9.1
Maternity Hospital	151	3.3
Al-Noor Specialist Hospital	3,307	69.7
*Severity*		
ICU	961	20.3
Non-ICU	3,781	79.7
*Gender*		
Male	3,162	66.7
Female	1,580	33.3
*Age (years)*		
<20	205	4.3
21-30	404	8.5
31-40	890	18.8
41-50	1,012	21.3
51-60	1,034	21.8
>60	1,197	25.2
*Nationality*		
Saudi	1,743	36.8
Myanmar	698	14.7
Bangladesh	447	9.4
Pakistan	380	8.0
Egypt	358	7.5
Yemen	302	6.4
India	223	4.7
Syria	70	1.5
Afghanistan	65	1.4
Nigeria	62	1.3
Sudan	57	1.2
Indonesia	58	1.2
Other	279	5.9
*BMI (kg/m^2^;n* = 1,236)		
<18.5 (underweight)	48	1.0
18.5–25 (normal)	544	11.5
25–30 (overweight)	437	9.2
>30 (obese)	207	4.4
*Patient Status*		
Dead	552	11.6
Discharged	3,401	71.7
Still admitted	789	16.6
*Diabetes*		
Yes	455	9.6
No	4,287	90.4
*Hypertension*		
Yes	328	6.9
No	4,414	93.1
*Heart diseases*		
Yes	51	1.1
No	4,691	98.9
*Other chronic diseases*		
Yes	102	2.2
No	4,640	97.8
LOSh (in Hospital) (median, IQR) (days)	4 (2-8)	
LOSi (in ICU) (median, IQR) (days)	4 (2-9)	

ICU: intensive care unit; BMI: body mass index; LOS: length of stay; IQR: interquartile range; Other chronic diseases: arthritis, asthma, back pain, cancer, chronic kidney disease, etc.; Heart diseases: coronary heart disease, cerebrovascular disease, peripheral arterial disease, rheumatic heart disease, congenital heart disease, and deep vein thrombosis.

RETRACTED

**Table 2:** Association between COVID-19 severity, LOS, and mortality with demographic variables.

Variables	ICU admission (severity)	LOSh	Death rate (mortality)
	*P* value	*P* value	*P* value
Gender	0.21	0.78	≤0.001
Age	≤0.001	≤0.001	≤0.001
Nationality	≤0.001	≤0.001	≤0.001
Body mass index	≤0.001	≤0.05	≤0.001
ICU admission (severity)	—	≤0.001	≤0.001
Death rate (mortality)	0.001	≤0.001	—
Diabetes	0.21	≤0.001	≤0.001
Hypertension	0.28	≤0.001	≤0.001
Heart diseases	≤0.05	0.33	≤0.001
Length of stay in hospital	≤0.001	—	≤0.001

## Data Availability

Data will be available on request.
